# MicroRNA-371-5p targets SOX2 in gastric cancer

**DOI:** 10.18632/oncotarget.8289

**Published:** 2016-03-23

**Authors:** Yu-Ji Li, Ming Dong, Fan-Min Kong, Jian-Ping Zhou, Dong Liang, Huan-Zhou Xue

**Affiliations:** ^1^ Department of General Surgery, The First Affiliated Hospital, China Medical University, Shenyang 110001, Liaoning, P.R. China

**Keywords:** microRNA-371-5p, gastric cancer, SOX2, diological significance

## Abstract

We evaluated miR-371-5p expression in gastric cancer (GC) tissues and its influence on the expression of downstream genes, especially *SOX2*. MiR-371-5p expression (measured using qRT-PCR) was upregulated in GC tissues and correlated positively with TNM staging and lymph node (LN) metastasis. MiR-371-5p expression was higher in human GC cell lines (AGS, MKN-28, BGC-823, MGC-803, SGC-7901 and MKN-45) than in human normal gastric epithelial (GES-1) cells (all *P* < 0.05). MGC-803 tumor cell growth (measured with an MTT assay), migration, and invasion (measured with Transwell chamber assays) were severely inhibited in cells transfected with a miR-371-5p inhibitor, whereas they were stimulated in cells transfected with SOX2 siRNA or miR-371-5p inhibitor + SOX2 siRNA. Expression of SOX2 mRNA and protein (assessed with qRT-PCR and Western blot) were greatly enhanced in the miR-371-5p inhibitor group. These results indicate that miR-371-5p expression is strongly upregulated in GC tissues and negatively correlated with SOX2 expression, while miR-371-5p expression is inversely related to proliferation, TNM stage, and LN metastasis of GC cells. Suppression of miR-371-5p may inhibit the growth and invasion of MGC-803 GC cells by upregulating SOX2 expression.

## INTRODUCTION

Gastric cancer (GC), also called stomach cancer, is the third leading cause of cancer death worldwide, with an estimated 700,000 deaths annually, accounting for 8.8% of total deaths globally in 2012 [1, 2]. GC is complex and multifactorial, and its carcinogenic mechanisms involve major exogenous factors, such as *Helicobacter pylori* infection, smoking, alcohol drinking, and habitual excessive salt intake [3–7]. Genetic and epigenetic alterations also contribute to the development of GC by causing the overexpression or hyperactivation of oncogenes and the loss of tumor suppressor genes [5, 8–11]. In this respect, biomarkers are important for the diagnosis and prediction of tumor behavior, and cancer-related microRNAs (miRs) have received significant attention recently for their relevance to the diagnosis and treatment of cancers, including GC [12–14].

Indeed, different miR expression profiles are observed in GC cells and normal control gastric epithelial cell ssues [15, 16], for instance, miR-371-5p, which belongs to the miR-371 cluster (located within a 1050-bp region on chromosome 19), is overexpressed in hepatocellular carcinoma and probably regulates cell cycle progression. Similarly, miR-371-5p expression is upregulated in nasopharyngeal carcinoma, lupus nephritis and prostate cancer [17–21]. Importantly, serum levels of miR-371-5p were found to besignificantly elevated in GC patients, such that GC patients could be discriminated from controls with 75% sensitivity and 63.41% specificity. Thus, miR-371-5p could serve as a biomarker for GC diagnosis; however, the underlying biological significance of miR-371-5p in the development of GC still remains unknown [15]. SOX2 is an important transcriptional regulator of the cell cycle, cell proliferation and apoptosis. SOX2 is also a gastric differentiation marker, and is often downregulated in GC. In addition, KI-67 expression has been suggested as a valuable independent prognostic predictor of the survival of GC patients [22–25]. miR-126 was over-expressed in GC and targeted SOX2, therefore, up-regulation of miR-126 inhibited SOX2 expression and promoted gastric carcinogenesis [29]. Notably, miR-371-5p is also overexpressed in colorectal cancer and down-regulated SOX2 expression, showing that Recently, *SOX2* was identified as a target gene inhibited by miR-371-5p; in this manner, miR-371-5p promotes cell proliferation, invasion, and epithelial-mesenchymal transition in colorectal cancer (CRC) [26].

We were interested in determining the biological mechanisms and significance of miR-371-5p in the development of GC. Thus, we investigated miR-371-5p expression in GC tissue and adjacent normal tissues.

## RESULTS

### Comparison of miR-371-5p expression in GC tissues and cells

MiR-371-5p expression in GC tissues and cells was evaluated by qRT-PCR. The results illustrated in Figure 1 clearly demonstrate the fluorescence background signal (baseline phase), exponential amplification of fluorescence (logarithmic growth) and stable amplification of fluorescence (stationary phase) for the amplification curves of miR-371-5p and U6 snRNA (Figure 1A). Furthermore, there were no signs of non-specific dissolution peak or miscellaneous peaks in the dissolution curves, which indicated the high specificity of the primer s and confirmed the absence of non-specific amplification products (Figure 1B).

**Figure 1:** (**A**) Amplification curves from qRT-PCR analysis of miR-371-5p and U6. (**B**) Dissolution curves of miR-371-5p after amplification. (**C**) Relative expression (median and interquartile range) of miRNA-371-5p in GC tissues and adjacent normal tissues. ΔCT was calculated as (CT miRNA-371-5p) - (CT U6 snRNA). *P < 0.05. (**D**) Relative expression (mean ± SD) of miRNA-371-5p in human GC cell lines (AGS, MKN-28, BGC-823, MGC-803, SGC-7901 and MKN-45) compared with human normal gastric epithelial cells (GES-1); all *P* < 0.05. qRT-PCR, quantitative real-time PCR; GC, gastric cancer.

The relative miR-371-5p expression in GC tissue and adjacent normal tissue was compared with a non-parametric rank test. MiR-371-5p expression was significantly greater in GC tissue than in adjacent normal tissue (*P* 0.007, Figure 1C). The relationships between relative miR-371-5p expression and clinicopathological features of GC are summarized in Table 1. The expression of miR-371-5p was markedly lower in GC patients with TNM I-II staging (0.17 [0.09–1.23]) than in those with III-IV staging (0.75 [0.30–2.32]) (*P* = 0.007). In addition, miR-371-5p expression was positively associated with LN metastasis in GC (*P* = 0.022). However, miR-371-5p expression was not related to age, sex, tumor location, or degree of differentiation in the GC samples (*P* = 0.276, *P* = 0.773, *P* = 0.870, *P* = 0.424, respectively).

**Table 1:** MiR-371-5p relative expressions in different clinicopathological characteristics of GC

Clinical and pathological data	Case number	miR-371-5p relative expression (2^−ΔΔCT^)	*Z* value	*P* value
Age (year)				
< 60	28	0.49 (0.10–1.71)	−1.089	0.276
≥ 60	32	0.44 (0.15–2.56)		
Sex				
male	29	0.58 (0.14–2.01)	−0.726	0.773
female	31	0.38 (0.11–2.27)		
Tumor location				
Near the pylorus	33	0.51 (0.14–2.10)	−0.163	0.870
Near the cardia	27	0.35 (0.13–2.06)		
Differentiation degree				
moderately to well differentiated	36	0.49 (0.13–1.29)	0.800	0.424
Poorly to non-differentiated	24	0.35 (0.12–1.97)		
LNM				
without metastasis	33	0.19 (0.09–1.16)	−2.290	0.022
with metastasis	27	0.69 (0.27–2.23)		
TNM staging				
I/II staging	30	0.17 (0.09–1.23)	−2.698	0.007
III/IV staging	30	0.75 (0.30–2.32)		

GC, gastric cancer.

The expression of miR-371-5p was then evaluated in GC cell lines and normal gastric epithelial cells. The results were compared by univariate ANOVA, followed by an LSD-*t* test for post hoc analysis (Figure 1D). MiR-371-5p expression was significantly higher in the human GC cell lines AGS, MKN-28, BGC-823, MGC-803, SGC-7901 and MKN-45 than in GES-1 normal human gastric epithelial cells (*P* = 0.003, *P* = 0.0002, *P* = 0.003, *P* = 0.0009, *P* = 0.005, *P* = 0.014). The highest level of miR-371-5p was detected in the MGC-803 cell line, which was thus selected for further investigation.

### Confirmation of SOX2 as the target gene of miR-371-5p

A bioinformatic analysis was conducted with TargetScan to predict the binding site of miR-371-5p in the 3′-untranslated region (3′-UTR) of *SOX2* (Figure 2A). As a test of the functionality of the predicted miR-371-5p-binding sites, 3′-UTR segments harboring the wild-type or mutant candidate motifs targeted by miR-371-5p were synthesized and sub-cloned into luciferase reporter vectors. The recombinant plasmids (Wt-miR-371-5p/SOX2 and Mut-miR-371-5p/SOX2) were co-transfected with miR-371-5p mimics, and the ability of miR-371-5p to bind to the 3′-UTR of *SOX2* was evaluated in luciferase assays The miR-371-5p mimics had no obvious effects on the luciferase activity of Mut-miR-371-5p/SOX2, but significantly reduced the luciferase activity (65%) of Wt-miR-371-5p/SOX2 (*P* = 1.482E-10, Figure 2B).

**Figure 2:** *SOX2* is directly targeted by miR-371-5p (**A**) MiR-371-5p target site in the 3′-UTR of *SOX2*. (**B**) Luciferase assays were used to evaluate the ability of miR-371-5p to bind to the 3′-UTR of *SOX2*. Wt-miR-371-5p/SOX2 or Mut-miR-371-5p/SOX2 was co-transfected with miR-371-5p mimics. *P < 0.05, miR-371-5p mimic vs. negative control.

### Comparison between SOX2 and KI-67 expression in GC and adjacent normal tissues

Immunohistochemistry analyses of SOX2 and KI-67 expression were performed on GC tissues and adjacent normal tissues, and χ^2^ tests were used to compare the expression of these proteins between the two tissue types. Strong staining of SOX2 was visible as a yellowish-brown granular or diffuse staining pattern, mainly in the cytoplasm of GC tissues (Figure 3A). Positive expression of SOX2 was detected in 26.67% (16/60) of GC tissues, a markedly lower proportion than in the adjacent normal tissues (75%, 45/60, *P* = 1.188E-7, Table 2). In GC tissues, KI-67 was mainly localized to the nuclei, where it was visible as brownish-yellow staining (Figure 3B). The immunoreactivity and histological appearance indicated that KI-67 protein expression occurred more frequently in GC tissues (58.33%, 35/60) than in the adjacent normal tissues (16.67%, 10/60, *P* = 2.428E-6, Table 2).

**Figure 3:** (**A**) SOX2 expression in GC tissues relative to adjacent normal tissues (200×). Strong staining of SOX2 is mainly visible in the cytoplasm as a yellowish-brown granular or diffuse staining pattern. SOX2 expression was markedly lower in GC tissues than in the adjacent normal tissues. (**B**) KI-67 expression in GC tissues relative to adjacent normal tissues (200×). KI-67 was mainly localized to the nuclei in GC tissues; it appears brownish-yellow in color. KI-67 protein was more frequently detected in GC tissues than in the adjacent normal tissues. GC, gastric cancer.

**Table 2:** SOX2 and Ki-67 expressions in gastric cancer tissues and adjacent normal tissues

Protein expression		GC tissues	Adjacent tissues	*χ*^2^ value	*P*
SOX2	+	9	11	33.22	1.188E-7
	++	5	15		
	+++	2	19		
	−	44	15		
Ki-67	+	8	6	26.27	2.428E-6
	++	12	3		
	+++	15	1		
	−	25	50		

GC, gastric cancer.

### Comparison of SOX2 expression among GC tissues with different characteristics

The associations of SOX2 expression with clinicopathological characteristics of GC were then evaluated with χ^2^ tests (Table 3). SOX2 expression was significantly lower in GC tissues with LN metastasis than in those without LN metastasis (3.70% vs. 45.45%, *P* = 2.745E-4). In addition, SOX2 expression was significantly lower in poorly differentiated and undifferentiated GC tissues than in well-differentiated or moderately differentiated GC tissues (8.33% vs. 38.89%, *P* = 0.015). Further, significantly higher SOX2 expression was observed in GC patients with TNM I/II staging than in those with III/IV staging (46.67% vs. 6.67%, *P* = 4.596E-4). However, no association was found between SOX2 expression and age, sex or tumor location in GC patients (all *P* > 0.05).

**Table 3:** SOX2 expressions and clinicopathological characteristics of GC

Clinical and pathological data	Case number	SOX2		Positive rate (%)	*P*
		Negative	Positive		
Age (year)					
< 60	28	19	9	32.14	0.397
≥ 60	32	25	7	21.88	
Sex					
male	29	23	6	20.69	0.387
female	31	21	10	32.26	
Tumor location					
Near the pylorus	33	25	8	24.24	0.771
Near the cardia	27	19	8	29.63	
Differentiation degree					
Moderately to well differentiated	36	22	14	38.89	0.015
Poorly to non-differentiated	24	22	2	8.33	
LNM					
without metastasis	33	18	15	45.45	2.745E-4
with metastasis	27	26	1	3.70	
TNM staging					
I/II staging	30	16	14	46.67	4.596E-4
III/IV staging	30	28	2	6.67	

GC, gastric cancer.

### Correlation analysis

The correlation of miR-371-5p expression with the expression of SOX2 and KI-67 in GC tissue was calculated with the nonparametric Spearman's rank test (Table 4). MiR-371-5p expression negatively correlated with SOX2 expression in GC tissues (*r* = −0.677, *P* = 1.050E-8). However, no association between miR-371-5p expression and KI-67 expression was observed (*r* = 0.178, *P* = 0.554). KI-67 expression also negatively correlated with SOX2 expression in GC tissues (*r* = −0.621, *P* = 0.005).

**Table 4:** Association of miR-371-5p expressions with SOX2 and Ki-67 expressions in GC tissues

	microRNA-371-5p	SOX2	Ki-67
microRNA-371-5p	1.000	−0.677^a^	0.178^b^
SOX2	−0. 677^a^	1.000	−0.621^c^
Ki-67	0.178^b^	−0.621^c^	1.000

Note: r, correlation coefficient of the Spearman analysis;

a the correlation of microRNA-371-5p and SOX2 expression levels, P < 0.001;

b the correlation of microRNA-371-5p and Ki-67 expression levels, P = 0.554;

c the correlation of SOX2 and Ki-67 expression levels, P = 0.005.

### MTT assay

The effect of inhibiting miR-371-5p expression on GC cell growth was measured with an MTT assay in cells transfected with a miR-371-5p inhibitor, SOX2 siRNA, or both (Figure 4). OD values were compared among different time points and groups by univariate ANOVA, followed by an LSD-*t* test for post hoc analysis. Twenty-four hours after transfection, tumor growth was greatly inhibited (*P* < 0.05) in the miR-371-5p inhibitor group relative to the blank control and NC groups, indicating that low expression of miR-371-5p could suppress GC cell growth. Furthermore, the OD values at 24, 48, 72 and 96 h post-transfection in the SOX2 siRNA group and the miR-371-5p inhibitor + SOX2 siRNA group were significantly greater than those in the blank control and NC groups (all *P* < 0.05).

**Figure 4:** MTT assay detecting the effect of inhibiting miR-371-5p expression on GC cell growth (compared to the control group, *P* < 0.05) GC, gastric cancer.

### Transwell chamber assay: migration ability of gastric cells

An *in vitro* Transwell chamber assay was performed to determine the effect of inhibiting miR-371-5p expression on the migration ability of gastric cells (Figure 5). The numbers of migrating cells among the different transfection groups were compared by univariate ANOVA, followed by an LSD-*t* test for post hoc analysis. Using an *in vitro* transwell migration assay (Figure 5), results demonstrated that the number of cells that migrated through the polycarbonate membrane to the lower surface of the membrane 48 h after culture did not differ between the blank control group and the NC group (75.3 ± 2.5 vs. 71.3 ± 2.1, *P* = 0.516). On the other hand, the number of cells that migrated to the lower surface of the membrane was 39.7 ± 2.5 in the miR-371-5p inhibitor group, significantly lower than that in the blank control group or the NC group (*P* = 1.603E-8 and *P* = 2.189E-8). Thus, exogenous inhibition of miR-371-5p expression impaired the migration ability of MGC-803 cells.

**Figure 5:** Transwell chamber assay exploring the effect of miR-371-5p inhibitor transfection on the migration ability of MGC-803 cells (200×) (**A**) Blank control group; (**B**) NC group; (**C**) miR-371-5p inhibitor group; (**D**) SOX2 siRNA group; (**E**) miR-371-5p inhibitor + SOX2 siRNA group; (**F**) corresponding histogram of the Transwell migration of MGC-803 cells after transfection. Cell migration was measured with normal Transwell chambers and expressed as the migration index (%). The values represent the mean ± SD, and a *P* value of < 0.05 was considered statistically significant. NC, negative control; *P < 0.05 compared with the blank control group and the NC group ^#^*P* < 0.05 compared with the miR-371-5p inhibitor group.

Further, the number of migrated cells was significantly higher in the SOX2 siRNA group (101.0 ± 4.0) than in the blank control group (75.3 ± 2.5, *P* = 1.910E-6) or the NC group (71.3 ± 2.1, *P* = 4.506E-7). The number of cells that migrated through the polycarbonate membrane was greater in the miR-371-5p inhibitor + SOX2 siRNA group than in the miR-371-5p inhibitor group (83.7 ± 3.1 vs. 39.7 ± 2.5, *P* = 7.701E-9). Thus, exogenous inhibition of *SOX2* appears to promote the migration of MGC-803 cells, as SOX2 siRNA restored the migration ability that had been impaired by the miR-371-5p inhibitor.

### Transwell chamber assay: basement membrane penetration of gastric cells

An additional Transwell chamber assay was performed to determine the effect of inhibiting miR-371-5p expression on the ability of gastric cells to penetrate the basement membrane (Figure 6). The numbers of penetrating cells among the different transfection groups were compared by univariate ANOVA, followed by an LSD-*t* test for post hoc analysis. Transwell chamber result (Figure 6) suggested that the number of cells that penetrated through the polycarbonate membrane to the lower surface of the membrane in the miR-371-5p inhibitor group (33.7 ± 2.5) was significantly lower than that of the blank control group (58.3 ± 1.5, *P* = 6.438E-8) or the NC group (56.7 ± 2.1, *P* = 2.636E-7) There was no significant difference in the number of invasive cells between the blank control group and the NC group (*P* = 0.203). Thus, reduced miR-371-5p expression appeared to inhibit the invasion ability of MGC-803 cells. Additionally, the number of invasive cells was significantly higher in the SOX2 siRNA group (73.0 ± 3.6) and in the miR-371-5p inhibitor + SOX2 siRNA group (69.3 ± 2.5) than in the blank control group (*P* = 2.994E-5, *P* = 8.330E-5 and *P* = 2.973E-5, *P* = 2.522E-5). Thus, exogenous reduction of *SOX2* expression seems to promote the invasion of MGC-803 cells, as SOX2 siRNA restored the invasion ability that had been impaired by the miR-371-5p inhibitor.

**Figure 6:** Transwell chamber assay exploring the effect of miR-371-5p inhibitor transfection on the invasion ability of MGC-803 cells (200×) (**A**) Blank control group; (**B**) NC group; (**C**) miR-371-5p inhibitor group; (**D**) SOX2 siRNA group; (**E**) miR-371-5p inhibitor + SOX2 siRNA group; (**F**) corresponding histogram of Transwell invasion of MGC-803 cells after transfection. Cell invasion was measured with Matrigel-coated Transwell chambers and expressed as the invasion index (%). The values represent the mean ± SD, and a *P* value of < 0.05 was considered statistically significant. NC, negative control; *P < 0.05 compared with the blank control group and the NC group ^#^*P* < 0.05 compared with the miR-371-5p inhibitor group.

### Determination of SOX2 mRNA levels in transfected cells

Fluorescence-based qRT-PCR analysis of *SOX2* mRNA expression was also conducted on the aforementioned transfected cell lines (Figure 7A). *SOX2* mRNA levels among the different groups were compared by univariate ANOVA, followed by an LSD-*t* test for post hoc analysis. The *SOX2* mRNA level was higher in the miR-371-5p inhibitor group than in the blank control and NC groups (*P* = 1.103E-11, *P* = 7.182E-11, respectively), while no difference was found between the blank control group and the NC group (*P* = 0.108). Further, the *SOX2* mRNA level was significantly lower in the SOX2 siRNA group and the miR-371-5p inhibitor + SOX2 siRNA group than in the blank control group and the NC group (*P* = 1.242E-8, *P* = 2.474E-7 and *P* = 1.618E-7, *P* = 9.123E-7).

**Figure 7:** (**A**) Determination of *SOX2* mRNA levels by fluorescence-based qRT-PCR. (**B**) Quantitative determination of SOX2 expression by Western Blotting after miR-371-5p inhibitor transfection. qRT-PCR, quantitative real-time PCR; *P < 0.05 compared with the blank control group and the NC group ^#^*P* < 0.05 compared with the miR-371-5p inhibitor group.

### Determination of SOX2 protein levels in transfected cells

SOX2 protein expression in the transfected cell lines was then assessed by Western Blot (Figure 7B). The SOX2 levels among the different groups were compared by univariate ANOVA, followed by an LSD-*t* test for post hoc analysis. Twenty-four hours after the transfection of gastric MGC-803 cells with the miR-371-5p inhibitor, SOX2 expression was upregulated relative to the control groups (*P* = 3.791E-9, *P* = 2.139E-8). Further, the expression of SOX2 was significantly lower in the SOX2 siRNA group and the miR-371-5p inhibitor + SOX2 siRNA group than in the blank control group and the NC group (*P* = 5.313E-11, *P* = 1.143E-7 and *P* = 4.005E-9, *P* = 1.004E-6, while there was no difference between the blank control group and the NC group (*P* = 0.235).

## DISCUSSION

Our main objective was to understand the biological significance of miR-371-5p in the development of GC. In the current study, miR-371-5p expression was higher in GC tissues than in the adjacent normal tissues. In addition, higher expression of miR-371-5p was observed in patients with TNM stage III–IV and positive LN metastasis than in their respective controls, suggesting that miR-371-5p may promote the progression of GC. Furthermore, miR-371-5p was highly expressed in human GC cell lines (AGS, MKN-28, BGC-823, MGC-803, SGC-7901 and MKN-45) relative to GES-1 normal human gastric epithelial cells. Among these cell lines, the highest expression of miR-371-5p was observed in MGC-803 cells, so this cell line was selected for the subsequent *in vitro* investigations.

A previous study demonstrated that miR-371-5p downregulated *PRPF4B* mRNA and thus facilitated cell cycle progression in human hepatocellular carcinoma [18]. Our study revealed that *SOX2* may also be a downstream target of miR-371-5p and thus participate in GC pathogenesis. Indeed, high expression of SOX2 promotes the differentiation of stomach epithelial cells into mature cells, while low expression of SOX2 can cause the continual division of epithelial cells, indicating that SOX2 is crucial for gastric tumor suppression [22, 27]. In the present study, immunohistochemistry analysis further confirmed that SOX2 expression was markedly lower in GC tissues than in the adjacent normal tissues. Overexpression of SOX2 was suggested to be negatively linked to LN metastasis and tumor invasion stage in GC by repressing placenta-specific protein 1 expression [28].

In this study, KI-67 expression was also greater in GC tissues than in adjacent normal tissues. The high expression of KI-67 antigen in GC tissues was strong evidence of the rapid proliferation and aggressiveness of gastric malignancies. Further, overexpression of KI-67 correlated with low expression of SOX2 in the GC tissues, which further supported the involvement of SOX2 in GC development, and hinted that SOX2 might be a target of miR-371-5p.

Having established miR-371-5p as an onco-promoter in GC and identified the potential function of SOX2 in GC, we next investigated the possible relationship of miR-371-5p and SOX2 in GC progression. Notably, defects in cell cycle control promote tumor proliferation and growth; thus, we first considered whether miR-371-5p might promote tumor growth by targeting SOX2 [29]. With respect to the specific relationship between miR-371-5p and SOX2, we hypothesized that miR-371-5p expression would inversely correlate with SOX2 expression in C patients. The results of our MTT, Transwell chamber and qRT-PCR assays suggested that the inhibition f miR-371-5p expression significantly suppressed MGC-803 cell growth, metastasis, and invasion. The Western Blotting results further testified that SOX2 was directly negatively regulated by miR-371-5p. Thus, we conclude that suppression of miR-371-5p inhibited tumor cell proliferation, metastasis and invasion by releasing the suppression of SOX2. In partial agreement with our study, Zhang *et al.* also found that SOX2 expression inversely correlated with GC prognosis, and that low SOX2 expression was associated with tumor metastasis [30]. Li and colleagues went one step further and identified a negative association between miR-371-5p and SOX2 expression in CRC cell lines and tissues [26]. Both GC and CRC are digestive tract tumors, so these previous CRC data may support the results of our current investigation. At the same time, the present paucity of research on this subject highlights the significance of our identification of the relationships among miR-371-5p, SOX2, and GC.

In summary, we demonstrated that miR-371-5p expression was highly upregulated in GC tissues and negatively correlated with SOX2 expression. Meanwhile, there was an inverse relationship between SOX2 expression and the cell proliferation, TNM stage, and LN metastasis of GC tissues. Further, suppression of miR-371-5p expression appeared to inhibit the growth and invasion of GC MGC-803 cells by upregulating SOX2 expression. Thus miR-371-5p can be used as an effective oncogenic biomarker for the screening of high-risk populations, as well as a therapeutic target in GC treatment.

## MATERIALS AND METHODS

### Ethics statement

The study conformed to the guidelines of the research ethics committee at the First Affiliated Hospital, China Medical University. All experimental protocols were approved by the research ethics committee at the First Affiliated Hospital. All aspects of the current study complied with the World Medical Association Declaration of Helsinki [31]. Institutional review board (IRB) approval and written informed consent from all patients were obtained prior to surgery.

### Patients and tissue specimens

Samples of tumor tissue and adjacent normal tissue (about 5 cm away from the primary tumor margin) were collected from 60 GC patients (29 males, 31 females, average age: 57.5 ± 14.2 years) undergoing surgical resections at the Department of Gastrointestinal Surgery of The People's Hospital of Zhengzhou University between August 2012 and October 2012. Tumor samples were classified in accordance with the TNM (2010) classification criteria of the Union for International Cancer Control (UICC) and were reviewed independently by two pathologists [32]. Of the 60 GC tissues, 36 GC specimens were well- or moderately differentiated, while the remaining 24 GC specimens were poorly-differentiated or undifferentiated. Based on TNM staging, 30 of the 60 GC tissues were classified as TNM stage III–IV, while the other 30 specimens were classified as TNM stage I–II Twenty-seven GC tissues had lymph node (LN) metastasis, while 33 did not. None of the patients had received any preoperative treatment, including radiation therapy, chemotherapy or non-steroidal anti-inflammatory drugs. GC samples and adjacent normal tissues were cut into two parts after surgical removal. Half of each tissue was frozen immediately in liquid nitrogen and stored at −80°C, while the other half was paraffin-embedded after formalin fixation.

### Cell culture

Human GC cell lines (AGS, MKN-28, BGC-823, MGC-803, SGC-7901 and MKN-45) and human normal gastric epithelial cells (GES-1) were purchased from the Cell bank of the Chinese Academy of Sciences, Shanghai and from the human tumor cell bank at the Institute for Cancer Research, Peking Union Medical College Hospital. Cells were incubated in RPMI-1640 medium supplemented with 10% fetal calf serum (5% CO_2_, 37°C, humidity 95%). The cell cultures were maintained in monolayer and passaged when they reached 90% confluence. The medium was removed and cells were washed twice in PBS. Then, cells were digested with 0.25% trypsin, which was removed after dilatation of the intercellular spaces was observed. A single cell suspension was prepared by constant pipetting and the cell culture was passaged in RPMI-1640 medium supplemented with 10% fetal calf serum.

### RNA extraction and quantitative real-time PCR (qRT-PCR)

qRT-PCR was used to quantify miRNA-371-5p expression in GC tissues and cell lines. Total RNA was isolated from gastric tissues with the Genolution miRNA purification kit (Day root Biotechnology Co. Ltd., Beijing, China) in accordance with the manufacturer's instructions. U6 small nuclear RNA (snRNA) was used as a normalization control. The qRT-PCR reaction was carried out with the miRCURY LNA^™^ SYBR^®^ Green master mix Universal (Exiqon) on an ABI 6000 Real-Time PCR System. PCR programs were performed under the following conditions: denaturation at 95°C for 10 min, followed by 40 cycles of 95°C for 10 s and 60°C for 1 min. The primers used for qRT-PCR were as follows: miR-371-5p primer: 5′-ACTCAAACTGTGGGGGCA-3′, U6 snRNA primer: 5′-TTCGTGAAGCGTTCCATATTTT-3′. The relative expression of miRNA-371-5p was calculated by the 2−ΔΔCt method, where ΔCT is calculated as (CT miRNA-371-5p) - (CT U6 snRNA), and ΔΔCT is calculated as (ΔCT cancer) - (Δ CT control).

### Luciferase reporter gene assay

For the construction of a luciferase reporter vector, DNA was extracted with the TIANamp Genomic DNA Kit (Tiangen, China) with strict adherence to the manufacturer's instructions. A Dual-luciferase reporter vector construction was designed with Primer Premier 5.0 (Premier Biosoft, USA). The specific primers were: SOX2-3′UTR: Wt: Forward: 5′-GCGGCATCTCGAGCAAAAGAGGAGAGTAAGAAACAGC A-3′, Reverse: 5′-TATAGCGGCCGCCATGGATTC TCGGCAGACTGATTCA-3′; Mut: Forward 5′-TGACG CGTATCGAGATAAACATGGCAATC-3′, Reverse: 5′-TA CAAAAGTTGCTTGCAAATATTAAAACAT-3′. The luciferase activities of the tissue samples were measured with the Dual-Luciferase Reporter Assay system (Promega, Cat. # E1910). Forty-eight hours after transfection, the old medium was aspirated and the cells were washed twice in PBS. The transfected cells were lysed in 100 μL of passive lysis buffer (Promega) and gently agitated at room temperature for 15 minutes; then, the cell lysate was collected. Vigor testing was completed in 10 seconds with a 2-second delay initially. For the measurement of firefly luciferase activity, 100 μL Luciferase Assay Reagent II (LAR II, Stratagene) and Stop & Glo™ (LAR II Stop & Glo™, Stratagene) Reagent were added to 20 μL of the harvested cell lysate.

### Immunohistochemistry (IHC) staining

Tissues were cut into 4-μm-thick sections and incubated for 30 min with 3% hydrogen peroxide to eliminate endogenous peroxidase activity. Then, the sections were washed and incubated with rabbit monoclonal SOX2 (1:300, Boosen Biotechnology Co., Ltd., Beijing, China) and mouse monoclonal KI-67 (Maixin Biotechnology Co., Ltd., Fuzhou, China) overnight at 4°C. The sections were added with polymerase auxiliary agent for incubation for 20 min in room temperature. After the sections were incubated for 30 min with peroxidase-labeled goat anti-rabbit antibodies (secondary antibodies) at room temperature, nuclei were counterstained by the avidin-biotin technique with 3, 3′-diaminobenzidine tetrahydrochloride (DAB) and hematoxylin for visualization. PBS was substituted for the primary antibody as a negative control. The expression of SOX2 and KI-67 (approved name: MKI67) was estimated by semi-quantitative analysis. SOX2-positive cells were identified as those with brown granules in the cytoplasm and on the cell membrane, while KI-67-positive cells were identified as those with brown granules in the nuclei. Five fields (×400) were randomly viewed at high magnification from each cancerous tissue (100 cells per field) and the number of positive tumor cells expressing SOX2 and KI-67 in each field was counted. The percentage of positive cells (positively-stained cells/total tumor cells × 100%) was calculated and denoted as follows: < 10% was considered as (−), 10–50% as (+), 51–80% as (++), and ≥ 81% as (+++).

### Transfection

Cultured cells were grouped into the following five groups: (1) the blank control group, without any transfection; (2) the negative control (NC) group, for which a NC plasmid of the miR-371-5p inhibitor was prepared (transfection density 40 μmol L^−1^); (3) the miR-371-5p inhibitor group, in which the miR-371-5p inhibitor (Shanghai GenePharma Co., Ltd) was used to reduce post-transfection expression of miR-371-5p; (4) the SOX2 siRNA group, transfected with SOX2 siRNA (Shanghai GenePharma Co., Ltd); and (5) the miR-371-5p inhibitor + SOX2 siRNA group, co-transfected with miR-371-5p inhibitor and SOX2 siRNA. The cells were inoculated into complete medium in a 50-mL flask at the appropriate cell density for transfection (30−50%). In a sterile centrifuge tube, a lipofectamin 2000 mixture was prepared (5 μL lipofectamin 2000 + 100 μL serum-free medium) and kept at room temperature for 5 mi. A DNA mixture (50 nmol siRNA + 100 μL serum-free medium) was prepared in a separate sterile tube, added to the lipofectamin 2000 mixture, and incubated at room temperature for 20 min to allow the formation of the DNA-liposome complex. Then, the cells in the 50-mL flask were washed in serum-free medium. Serum-free (antibiotic-free) medium was added to the DNA-liposome complex and mixed gently, and this mixture was added to the cells in the flask. The flask was incubated at 37°C with 5% CO_2_ for 6−8 h; then, the medium was replaced with complete medium. After 24- to 48-h incubation, all cells were collected for protein extraction.

### MTT assay

Transfected cells were cultured until 80% confluent and washed twice in PBS. Cells were digested with trypsin and a single cell suspension was prepared by pipetting. Cells were counted with a cell counter and inoculated into a 96-well plate (3−6×10^3^ cells [200 μL]/well, six wells per group). Cells were cultured for 24−72 h (37°C, 5% CO2) and then 20 μL of MTT solution (5 mg/mL, Sigma) was added to each well. The cells were then cultured for another 4 h (37°C, 5% CO_2_), and the medium was discarded. Next, 150 μL of DMSO was added to each well and the plate was gently shaken for 10 min to dissolve the crystals. The absorbance of each well was read after 12, 24, 48, 72 and 96 h on a microplate reader. The interval time was set as the abscissa and the absorbance value was set as the ordinate for the MTT curve. This experiment was repeated in triplicate.

### Measurement of cell migration and invasion in transwell chambers

(1) Cell migration assay: Normal chambers were chosen for the migration assay. Seventy-two hours after transfection, cells were collected for the preparation of a cell suspension. Then, cells were seeded in the upper chamber of a Transwell plate (Corning Incorporated, USA) and uniformly spread on the filter. All Transwell chambers were incubated at 37°C and 5% CO_2_ in culture medium for 48 h. The cells remaining on the upper surface of the filter were removed by gentle wiping with a cotton swab. Subsequently, the Transwell chambers were fixed in 95% ethanol for 15−20 min and washed in tap water. Eosin was added to each chamber for 10 min, after which the chambers were washed again in tap water. The chambers were inverted, dried, fixed with neutral balata, and observed and imaged on a high-power inverted microscope. Cells were then counted in five randomly chosen visual fields (200×) and the average value was calculated. The migration index (%) was calculated from the number of cells migrating through the polycarbonate membrane.

(2) Cell invasion assay: Matrigel-coated chambers were used for the invasion assay. To prepare Matrigel-coated plates, the Matrigel matrix was thawed overnight on ice at 4°C, diluted to 30 μL with serum-free DMEM medium (1:3), seeded three times into the upper well of a Transwell chamber containing a microporous membrane (15 μl, 7.5 μl, and 7.5 μl, respectively) with intervals of 10 min. The suspended cells were seeded in the upper chamber of the Transwell plate, and 0.5 mL of DMEM culture medium (with 10% fetal bovine serum) was then added to the lower chamber of the 24-well plate. The invasion index (%) was calculated from the number of cells that invaded through the Matrigel.

### Detection of SOX2 mRNA by fluorescence-based qRT-PCR

Total RNA was extracted from transfected cells with an RNAqueous kit (Ambion) in strict accordance with the manufacturer's instructions, and reverse transcribed with an iScript™ cDNA synthesis kit (Fermentas). The PCR reaction was quantified with a fluorometric DNA quantification kit (Fermentas). PCR primers were synthesized by Invitrogen, Guangzhou. The primer sequences for *SOX2* were as follows: upstream primer: 5′-CGAGATAAACATGGCAATCAAT-3′, downstream primer: 5′-ATTCAGCAAGAAGCCTCTCCTT-3′. *GAPDH* was used as an internal control; the primer sequences were: 5′-GTGGACCTGACCTGCGTCT-3′ (upstream primer), 5′-GGAGGAGTGGGTGTCGCTGT-3′ (downstream primer). The PCR cycle conditions were as follows: initial denaturation at 50°C for 2 min and 95°C for 10 min, followed by 40 cycles of 95°C for 15 s, 56°C for 45 s. The relative expression of *SOX2* was determined with the 2^−ΔΔCt^ method with *GAPDH* as a reference gene. Each specimen was tested in triplicate, and the entire experiment was repeated in triplicate with similar results.

### Western blotting for the expression of SOX2

The transfected cell cultures were washed three times in pre-cooled PBS. Then, the cells were lysed with a protein extraction lysate (100 μL/50-mL flask) and kept on ice for 30 min. The cells were centrifuged at 12,000 rpm for 10 min at 4°C and the supernatant was divided into 0.5-mL centrifuge tubes and stored at −20°C. Bovine serum albumin (BSA) standard (2 μg/μl) was diluted to 20 μg/μl, 15 μg/μl, 10 μg/μl, 5 μg/μl, 2.5 μg/μl and 0 μg/μl. Solution A and Solution B in BCA kit (Pierce) were prepared as 50:1 right after the dosage of BCA detection reagent was calculated. Lysed protein samples (2 μl) were diluted with 18 μl ddH2O and there were 2 wells of each sample. Detection solution (200 μl) was added into each well of 96 wells plate and 10 μl diluted standard/detected samples were then added into each well. The plate was shaken gently, incubated at 37°C for 30 min and cooled to room temperature. The absorbance of each sample was read at 490 nm through microplate reader. The standard curve was drawn and protein concentration of each sample was calculated. The samples were stored at −70°C for further analysis.

Electrophoresis was carried out in a cold chamber (4°C) for 1–2 h (stacking gel/40 V, separation gel/120 V). The electrophoresed proteins were transferred to a polyvinylidene fluoride (PVDF) membrane (4°C, 2 h), which was then soaked in TBST containing 5% skim milk and incubated for 1−2 h at room temperature. The membrane was incubated with SOX2 primary antibody (SUNBIO, Shanghai) overnight at 4°C, and then washed three times for 10 min with TBST. Next, mouse secondary antibody was added for a 1-h incubation at room temperature. Again, the membrane was washed three times for 10 min with TBST. The membrane was exposed to film with a chemiluminescent agent and the data were analyzed.

### Statistical analysis

All statistical analyses were performed with SPSS 18.0 software. The relative expression of miR-371-5p in GC tissues and adjacent normal tissues was expressed as the median (interquartile range) and analyzed by a non-parametric test, Wilcoxon's test. Other measurement data were expressed as mean ± standard deviation (SD). Univariate analysis of variance (ANOVA) was used for comparisons among multiple groups. Pairwise comparisons between groups were conducted with the LSD-*t* test for post hoc analysis. Categorical data were presented as ratios or percentages, and proportions were compared by χ^2^ tests. Correlations of miR-371-5p expression with the expression of SOX2 and KI-67 were calculated with the nonparametric Spearman's rank test. A *P* value < 0.05 was considered statistically significant.
